# Maintenance Therapy with Partially Hydrolyzed Guar Gum in the Conservative Treatment of Chronic Anal Fissure: Results of a Prospective, Randomized Study

**DOI:** 10.1155/2014/964942

**Published:** 2014-06-25

**Authors:** Antonio Brillantino, Francesca Iacobellis, Giuseppe Izzo, Natale Di Martino, Roberto Grassi, Adolfo Renzi

**Affiliations:** ^1^Surgery Department, Second University of Naples, Piazza Miraglia 2, 80138 Napoli, Italy; ^2^Radiology Department, Second University of Naples, Piazza Miraglia 2, 80138 Napoli, Italy; ^3^“Villa delle Querce” Hospital, Via Battistello Caracciolo 48, 80136 Napoli, Italy

## Abstract

*Purpose*. This study was designed to evaluate the role of maintenance therapy with partially hydrolyzed guar gum (PHGG) after topical application of glyceryl trinitrate (GTN) in the conservative treatment of chronic anal fissure (CAF). *Methods*. From all the patients with CAF observed during the study period, 165 subjects with healed CAF after standard therapy with topical GTN 0.4% ointment were randomized to receive (group II) or not (group I) maintenance therapy with PHGG for 10 months. Clinical and manometric followup was carried out 6 and 12 months after treatment. *Results*. At six-month followup, median visual analogue scale score was significantly higher in group I if compared with group II. The success and recurrence rate at 12-month followup were, respectively, 38.3% (28/73) in group I versus 58.5% (41/70) in group II (*P* = 0.019; Fisher's exact test) and 30.2% (13/43) in group I versus 14.5% (7/48) in group II (*P* = 0.0047; Fisher's exact test). *Conclusion*. The maintenance therapy with PHGG in patients with healed CAF after chemical sphincterotomy by topical application of GTN 0.4% ointment seems associated with a significant reduction of recurrence rate and with a significant increase of success rate at 12-month followup.

## 1. Introduction

Anal fissure is a common proctologic disease, characterized by an ulcer of anoderm, usually located in the posterior midline and extending from the dentate line to anal verge [1–3].

It represents the most common cause of severe anal pain and is associated with loss of working hours and reduced quality of life [4, 5].

The etiology of the chronic anal fissure (CAF) is still debated and has not been completely clarified, even if the increased anal tone and the mucosal ischemia resulting from internal sphincter spasm represent possible pathogenetic mechanisms [6–8].

Therefore, the principal therapeutic options are direct to decrease the anal canal pressure by means of surgical procedures (sphincter stretching, sphincterotomy) or local application of vasodilators [9–13].

Particularly, topical nitrates have been shown to reduce the anal sphincter hypertonia and have become, in many clinical contexts, the first-line pharmacological therapy for chronic anal fissure [6, 7, 9–11].

The role of fiber supplement in the conservative treatment of chronic anal fissure is still matter of debate.

Indeed, although the treatment of acute anal fissure with fiber supplement has been associated with increased healing rates, improvement of symptoms, and prevention of recurrence [14–16], in the chronic variety of fissure, this therapeutic approach is generally considered not effective [6] and the role of maintenance therapy with fibers, after conservative treatment with topical vasodilators, remains unclear.

This study was designed to evaluate the role of maintenance therapy with partially hydrolyzed guar gum in patients with healed CAF after conservative treatment with topical application of 0.4% glyceryl trinitrate (GTN) ointment.

## 2. Methods

### 2.1. Study Population

Between January 2008 and December 2011 all the patients with CAF (not healing in at least 6 weeks, keratinous edges, fibers of the internal anal sphincter visible, sentinel node, or hypertrophied anal papillae present) were considered for the enrollment in this prospective study.

All the patients underwent clinical evaluation, physical examination, colonoscopy, anorectal manometry, and evaluation of anal pain intensity by means of a 10-point visual analogue scale (VAS) [17].

Exclusion criteria included acute anal fissure, coexisting Crohn's disease or ulcerative colitis, TBC, HIV, pelvic radiotherapy or anorectal malignancies, anal incontinence, and previous treatment with topical vasodilators.

After clinical assessment, all the patients underwent medical therapy with topical application of GTN 0.4% ointment every 12 hours for 6 weeks and received standardized advice to follow a high fibre diet.

At the end of treatment cycle, all the subjects had clinical assessment with physical examination, proctoscopy, and evaluation of VAS score for anal pain.

On the basis of this last evaluation, were included in this study the patients with age between 18 and 70 years, showing both resolution of symptoms and fissure healing after 6 weeks of medical therapy with topical application of GTN 0.4% ointment, and available for short-term followup.

All the included patients were randomly assigned to receive (group II) or not (group I) maintenance therapy with PHGG oral supplementation (5 g/die) for 10 months (7 cycles of four weeks spaced by 2-week interval times).

Clinical and manometric followup was carried out 6 and 12 months after treatment. At each follow-up point, the assessment of pain by VAS scale was also performed.

The primary end points of the study were the success and recurrence rate at 12-month followup. The treatment strategy was considered successful when the resolution of symptoms and the disappearance of fissure on physical examination were simultaneously obtained.

The success and recurrence rate at 6-month followup and the adverse events to therapy constituted secondary end points.

All the patients with symptoms recurrence at 6- and 12-month followup were offered the opportunity to receive both prolonged medical and surgical therapy.

### 2.2. Anal Manometry

Anal manometry was performed using a silicone catheter with a diameter of 4.8 mm, provided with eight lumens and 4 radial openings located 5 cm from the tip and perfused with twice distilled water through a low-compliance pump, at a constant rate of 0.75 mL per minute with 1.2 kg/cm^2^ flow (Menfis Biomedica, Bologna, Italy). The catheter was connected to a personal computer via pressure transducers.

The lubricated catheter was introduced manually into the rectum, with patients in the left lateral decubitus position and flexed knees and hips.

The continuous pull-through technique was used with the catheter puller at a constant speed of 0.5 cm/s, for the evaluation of anal canal length (ACL), high pressure zone (HPZ), and mean resting pressure (MRP). The mean squeeze pressure (MSP) was recorded by means of the stationary pull-through technique.

Each investigation was repeated 3 times, and the mean value was taken as the result.

The same manometric procedure was performed in a control group including 22 normal volunteers: 11 women and 11 men (mean age: 44 years; range: 18–64 years).

### 2.3. Randomization and Blinding

The randomization list was computer-generated, with block size varying from 4 to 6 patients, and the list was maintained at the study center in sequentially numbered opaque envelopes. Patients were randomly assigned by extracting the next envelope in the sequence.

All researchers involved in data collection and analysis were blinded to the assigned treatment strategy.

### 2.4. Sample Size and Statistical Method

A retrospective analysis of clinical outcome in patients who underwent conservative treatment with topical 0.4% glyceryl trinitrate suggested 60% and 40% success rate, respectively, at 6- and 12-month followup. We hypothesized that a 60% success rate could be achieved in patients who underwent PHGG maintenance therapy at 12-month followup.

We estimated that 80 patients would be required in each group for the study to have a power of 80% to detect a difference of 20% age points in the success rates between the patients of the two groups at a significance level (alpha) of 0.05 (2-tailed test), if such a difference truly existed. We allowed for the possibility of incomplete data and included a total of 165 patients in this study.

The statistical analysis was carried out using the program InStat Graph-Pad Prism 5 (San Diego, California, USA).

Values are expressed as means ± standard deviation (SD) or medians (range). Continuous data were compared between each group using the Student *t*-test or the Mann-Whitney *U* test, when indicated.

Prevalence data were compared between groups using the Fisher's exact test.

A probability value of less than 0.05 was considered significant.

### 2.5. Ethics

The ethical committee of our institution approved the study protocol. All patients gave informed written consent.

## 3. Results

Among all the patients with CAF observed during the study period, 165 patients who satisfied selection criteria, were included in the study and randomized (Figure 1).

Among these last patients, 17 (9 in group I and 8 in group II) were lost to followup, whereas 5 group II patients (6.1%) interrupted treatment for the presence excessive flatulence and abdominal distension and were excluded from the study.

Overall, 143 (72.2%) patients [62 (43.3%) women and 81 (56.6%) men, median age 45 (range 19–68)] completed the entire followup and constituted the object of analysis.

No significant differences in patients' general features between the two groups were found (Table 1).

The most common preoperative symptom was anal pain, with a prevalence of 94.4% (135/143), whereas bleeding and constipation were reported, respectively, in 73.4% (105/143) and 55.9% (80/143) of cases.

Fifty (34.9%) patients (50/143) had chronic constipation whereas 30 (20.9%) showed constipation predominant irritable bowel syndrome according to Rome 3 criteria [18].

Baseline manometric data are summarized in Table 2. No significant differences in the manometric parameters between the patients of the two groups were found.

At manometry, mean anal resting pressure in patients with CAF was significantly higher than in the control group (100.01 ± 12.3 versus 66.8 ± 16.8 mm Hg; *P* < 0.0001: two-sample *t*-test).

At six-month followup the success rate was 58.9% (43/73) in group I and 68.5% (48/70) in group II (*P* = 0.29; Fisher's exact test), whereas recurrence rate was 41.09% (30/73) in group I and 31.4% (22/70) in group II (*P* = 0.29; Fisher's exact test) (Table 3).

Median VAS score was significantly higher in group I if compared with group II (3; 0–9 versus 2; 0–8: *P* = 0.03; Mann-Whitney *U* test).

All the 30 patients in group I and 22 patients in group II with symptoms recurrence at 6-month followup refused prolonged medical therapy and, consequently, underwent surgery.

The success and recurrence rate at 12-month followup were, respectively, 38.3% (28/73) in group I versus 58.5% (41/70) in group II (*P* = 0.019; Fisher's exact test) and 30.2% (13/43) in group I versus 14.5% (7/48) in group II (*P* = 0.0047; Fisher's exact test) (Table 3).

Overall, 12 months after standard therapy with topical nitrates, 43 (58.9%) group I and 29 (41.4%) group II patients with GTN-healed fissures experienced symptomatic recurrence (*P* = 0.045; Fischer's exact test).

All the patients with symptom recurrence after 1-year conservative treatment refused prolonged medical therapy and opted for surgery.

The adverse effects of PHGG dietary supplementation were abdominal distention and flatulence that were referred to by 23.4% (19/81) of treated patients. However, these symptoms caused interruption of treatment in 6.1% of cases.

## 4. Discussion

The chronic anal fissure is a common proctologic disease with unclear pathophysiology and variable treatment strategies ranging from conservative therapy (chemical or pharmacological sphincterotomy) to surgery.

The goal of treatment strategy is to decrease the anal resting pressure to interrupt the vicious cycle pain-spasm-ischemia involved in the arrest of fissure healing and self-maintaining of disease.

According to the literature, the conservative, medical therapy is considered the first-line treatment for CAF and can be based on topical application of 0.4% GTN [19–21].

However, with regards to healing, the therapeutic approach with topical nitrates seems marginally superior to placebo, achieving an overall response rate of about 55% and reporting a recurrence rate of approximately 50% [22].

One of the reasons of this high recurrence rate could be the transitory and reversible effect of topical nitrates in reducing muscle tone that, in presence of persistent microtrauma of the anoderm, caused by passage of fecal hard stool or diarrhea episodes, could not achieve stable fissure healing.

The role of fiber supplements in the management of anal fissure is still controversial.

Indeed, although the conservative therapeutic approach with fibers supplementation seems to achieve excellent results in the acute form of anal fissure, it is common opinion that fissures labeled as chronic or complicated neither heal spontaneously nor respond to this conservative therapy [5, 6].

Surprisingly, prospective studies concerning this question are lacking and the role of fiber supplement in the maintenance therapy of chronic anal fissure after chemical sphincterotomy has never been evaluated.

This study was designed to evaluate the role of maintenance therapy with 5 g/die of PHGG for ten months in patients with healed chronic anal fissure after 6-weeks topical application of GTN 0.4%.

Partially hydrolyzed guar gum (PHGG) is a water-soluble, nongelling fiber that has provided therapeutic benefits in patients with constipation and irritable bowel syndrome, such as improvement of fecal consistence, normalization of bowel movements, alleviation of abdominal symptoms, and improvement of quality of life [22–24].

In the light of these observations, we hypothesized that maintenance therapy with PHGG in patients with GTN-healed chronic anal fissures could achieve improvement of short-term outcome and reduction of recurrences.

Interestingly, in our series, more than 50% of patients with CAF showed an intestinal disorder motility, represented by chronic constipation and constipation predominant irritable bowel syndrome. These data seem to suggest that, in a large percentage of patients with CAF, the reiterated microtrauma of anoderm could represent a relevant risk factor for fissure recurrence.

Moreover, in our study, the maintenance therapy with PHGG was associated with significant improvement of 6-month median VAS score, significant reduction of 12-month recurrence rate, and significant increase of success rate at 12-month followup.

These data emphasize the use of oral fiber supplementation as adjuvant therapy in CAF and suggest that maintenance therapy with PHGG, through the normalization of bowel movements and consequent decrease of anoderm traumatism, could improve the clinical outcome in a large percentage of patients with healed CAF after standard conservative treatment with topical application of nitrates.

However, in our study, 41.4% of patients with GTN-healed CAF experienced symptomatic recurrence despite receiving maintenance therapy with fibers.

Probably, as well as anoderm traumatism, multiple factors are involved in the complex chronic fissure pathophysiology.

Particularly, the insufficient anal sphincter stretchability, the associated perianal sepsis and the coexistent sentinel pile have been advocated as additional pathogenetic factors and could explain both recurrences after conservative treatment and differences between surgical and pharmacological sphincterotomy outcome [5, 25, 26].

The optimal duration of conservative treatment with GTN 0.4% in patients with CAF is still a matter of debate.

We do not know if further cycles of medical therapy with topical nitrates or a treatment longer than 6 weeks could achieve a better clinical outcome in our patients.

Anyway, in our study, all the patients with symptoms recurrence refused prolonged medical therapy and, therefore, further researchers are needed to answer this question.

In the same way, it is unclear if the contemporaneous employment of topical nitrates and PHGG dietary supplementation could be associated, as our results could suggest, with a further increase of the success rate and improvement of VAS score.

However, this goes beyond the purpose of this trial and may be the object of further studies.

Abdominal distension and flatulence represent potential negative effects of dietary fibers. However, in our study, the oral fiber supplementation with PHGG seemed well tolerated by the patients. Indeed, although flatulence and abdominal distention were reported by 23.4% of treated patients, these symptoms caused interruption of treatment only in 6% of cases.

## 5. Conclusion

In the patients with healed CAF, after standard conservative treatment with topical nitrates, the maintenance therapy with PHGG (5 g/die) for 10 months seems to significantly reduce the recurrence rate and significantly increase the success rate at 1-year followup. Further researches with larger series are needed to confirm these data.

## Figures and Tables

**Figure 1:** CONSORT flow diagram.

**Table 1:** Patients characteristics.

Patient characteristics	Group I	Group II
Patients	73	70
Gender (M/F)	40/30	41/32
Mean age (yrs)	45 (5.2)	45 (4.3)
Range of age	19–67	21–68

Values are expressed as number of patients and means with standard deviation in parentheses.

**Table 2:** Baseline manometric data of 143 analyzed patients (73 in group I and 70 in group II).

Manometric findings	Group I	Group II	*P* value^a^
Anal canal length (mm)	26.3 (5.0)	27.1 (8.4)	0.65
High pressure zone (mm)	18.1 (5.0)	19.2 (6.0)	0.43
Mean resting pressure (mmHg)	101.3 (13.9)	99.8 (10.9)	0.47
Mean squeeze pressure (mmHg)	123.6 (22.6)	120.0 (20.0)	0.51
Rectoanal inhibitor reflex (mL)	25.7 (2.2)	23.2 (2.5)	0.54
First initial sensation (mL)	25.9 (5.8)	27.1 (6.8)	0.46
Rectal capacity (mL)	219 (30.9)	211 (33.9)	0.33

Values are expressed as means with standard deviations in parentheses.

^a^Unpaired *t*-test.

**Table 3:** End points of the study in the two groups of patients.

End points	Group I	Group II	*P* value^a^
6-month recurrence rate	30 (41.09)	22 (31.4)	0.29

12-month recurrence rate	13 (30.2)	7 (14.5)	0.0047
12-month success rate	28 (38.3)	41 (58.5)	0.0019

Values are expressed as number of patients with percentages in parentheses.

^a^Fisher's exact test.
